# Tumor growth suppression by inhibiting both autophagy and STAT3 signaling in HNSCC

**DOI:** 10.18632/oncotarget.6294

**Published:** 2015-10-30

**Authors:** Teng-Fei Fan, Lin-Lin Bu, Wei-Ming Wang, Si-Rui Ma, Jian-Feng Liu, Wei-Wei Deng, Liang Mao, Guang-Tao Yu, Cong-Fa Huang, Bing Liu, Wen-Feng Zhang, Zhi-Jun Sun

**Affiliations:** ^1^ The State Key Laboratory Breeding Base of Basic Science of Stomatology & Key Laboratory of Oral Biomedicine Ministry of Education, Wuhan University, Wuhan, China; ^2^ Department of Oral and Maxillofacial-Head and Neck Oncology, School and Hospital of Stomatology, Wuhan University, Wuhan, China

**Keywords:** autophagy, STAT3, head and neck cancer, apoptosis

## Abstract

Autophagy is considered as a double-edged sword. It can prolong the survival of cancer cells and enhance its resistance to apoptosis, and paradoxically, defective autophagy has been linked to increased tumorigenesis, but the mechanism behind this phenomenon is unclear. In this study, we demonstrated that decreased phosphorylation of signal transducer and activator of transcription 3 (*p*-STAT3) was correlated with increased autophagy through the Akt/mTOR and Erk signaling pathways in human head and neck squamous cell carcinoma (HNSCC). We also showed that blockage of STAT3 by NSC74859 could markedly induce apoptotic cell death and autophagy. Meanwhile, increased autophagy inhibited apoptosis. The pharmacological or genetic inhibition of autophagy and STAT3 further sensitized HNSCC cells to apoptosis. Furthermore, evidence from xenograft model proved that suppressed STAT3 activity combined with inhibition of autophagy promoted tumor regression better than either treatment alone. Taken together, this present study demonstrated that autophagy alleviates apoptotic cell death in HNSCC, and combination of inhibition of STAT3 by NSC74859 and autophagy might be a promising new therapeutic strategy for HNSCC.

## INTRODUCTION

Head and neck squamous cell carcinoma (HNSCC) represents a large heterogeneous group of tumors in the oral cavity, cheek, nasopharynx, oropharynx, hypopharynx, and larynx. The worldwide incidence of HNSCC exceeds 450,000 cases annually [1]. Intense research efforts have been carried out and considerable advances in HNSCC cancer therapy have been attained over the past decades; however, the survival rate of HNSCC patients has shown minimal improvement [2]. Mortality remains high because of therapy-resistant local recurrences and distant metastases. Thus, the development of potential alternative therapies and the discovery of novel mechanisms underlying HNSCC initiation and progression are necessary and urgent.

Apoptosis resistance, through which malignant cells evade cell death, is a hallmark of cancer cells [3]. Signal transducer and activator of transcription 3 (STAT3) plays key roles in this process [4]. STAT3 is constitutively activated in most malignant tumors [5–7], especially in HNSCC. Increasing evidence has indicated that STAT3 inhibition in cancer cell lines can trigger growth arrest or apoptosis [8–10]. Thus, STAT3 is a potential target in HNSCC therapy. Nonetheless, the underlying mechanism remains obscure. Blocking the phosphorylation of STAT3 (p-STAT3) potently stimulates the autophagic flux [11]. This finding indicates that autophagy is a novel mechanism by which HNSCC responds to STAT3 inhibition.

Autophagy is a cellular process of self-consumption in which bulk cytoplasm, long-lived proteins, and cellular organelles are engulfed into double-membrane vesicles termed autophagosomes and fuse with lysosomes, where the inner cargoes are degraded and recycled [12]. Autophagy helps tumor cells survive by conferring apoptosis resistance; inhibition of autophagy causes caspase-independent necrotic cell death, especially in the presence of other therapies [13]. However, whether or not all cancer cells show the same response to autophagy inhibition has yet to be determined. Understanding the interplay between apoptosis and autophagy in tumors is crucial to identify new targets for cancer therapy and improve therapeutic efficiency.

In the present study, we investigated the effect of blocking STAT3 signaling by NSC74859 (also known as S3I-201), an inhibitor of the dimerization and phosphorylation of STAT3. NSC74859 inhibited tumor growth by inducing apoptosis *in vitro* and *in vivo* in HNSCC. NSC74859 also induced autophagy, which was dependent on the Akt/mTOR and extracellular signal-regulated kinase (Erk) signaling pathways. Pharmacological or genetic inhibition of autophagy sensitized NSC74859-induced apoptosis in HNSCC. Our results provide molecular insights that the combination of autophagic and p-STAT3 inhibitors is a promising therapeutic strategy for HNSCC.

## RESULTS

### Blocking phosphorylation of STAT3 by NSC74859 induces HNSCC cell death

We investigated the effects of blocking STAT3 phosphorylation by NSC74859 (S3I-201) on apoptosis in HNSCC cell lines CAL27 and FaDu. Cultured CAL27 cells were treated with NSC74859 at increasing concentration. Hoechst nuclear staining was used to test cell apoptosis in NSC74859-treated HNSCC CAL27 cells; Figure 1A shows a positive staining of chromatin condensation. Treatment with NSC74859 increased TUNEL-positive cells in a dose-dependent manner (Supplementary Figure S1A). CAL27 cells were also analyzed by flow cytometry after Annexin V-FITC and PI dual labeling. As shown in Figure 1B, cells were treated with different concentration of NSC74859 for 24 h or 100 μM NSC74859 for 6, 12, and 24 h (Figures 1B and 1C). This treatment increased the percentage of apoptotic cells. Western blot analysis showed that the level of cleaved PARP (Cl-PARP) and cleaved-caspase 3 (Cl-casp3) increased with decreasing p-STAT3^T705^ expression; this effect was dose and time dependent (Figures 1D and 1E). To further demonstrate whether NSC74859-induced apoptosis in CAL27 cells was correlated to the activation of caspase3, a pan-caspase inhibitor benzyloxycarbonyl Val-Ala-Asp (O-methyl)-fluoro-methylketone (z-VAD-fmk) was employed. The results showed that when NSC74859 was combined with the treatment of 20 μM of z-VAD-fmk, the level of cleaved-PARP (Supplementary Figure S1B) and the apoptotic cells (Supplementary Figure S1C) were significantly decreased. These results reveal that NSC74859-induced apoptosis in CAL27 cells may partially depend on caspase 3 activation. The *in vitro* inhibition experiment was repeated in another cell line FaDu (Supplementary Figure S2). These results indicate that apoptosis is involved in the response of HNSCC to NSC74859 treatment.

**Figure 1:** Blocking phosphorylation of STAT3 by NSC74859 induces HNSCC cell death **A.** The morphologic changes of CAL27 treated with NSC74859 were captured using fluorescence microscopy with Hoechst 33258 staining. *Scale bar* 20 μm; **B.** CAL27 cells were treated with 50 μM, 100 μM, and 200 μM of NSC74859 for 24 h and stained with Annexin V/PI, then analyzed by flow cytometry. The percentages of Annexin V-positive cells were presented in bar charts; **C.** CAL27 cells were incubated with 100 μM of NSC74859 for 6, 12 and 24 h, then analyzed by flow cytometry. The percentages of Annexin V-positive cells were presented in bar charts; **P < 0.01. One-way ANOVA with post-Dunett analysis was used by GraphPad Prism5; **D.** CAL27 cells were treated with different concentration of NSC74859 for 24 h then western blot analysis was performed to assess the expression level of STAT3 and p-STAT3^T705^, cleaved-PARP (Cl-PARP) and cleaved-caspase 3(Cl-casp 3), GAPDH served as a loading control; Relative density data were calculated by Image J, and the data represented mean of three independent experiments. *P < 0.05, **P < 0.01; **E.** CAL27 cells were treated with 100 μM of NSC74859 for 6, 12 and 24 h then western blot analysis was performed to assess the expression level of STAT3 and p-STAT3^T705^, Cl-PARP and Cl-casp 3, GAPDH served as a loading control; Relative density data were calculated by Image J, and the data represented mean of three independent experiments. *P < 0.05, **P < 0.01, One-way ANOVA with post-Dunett analysis was used by GraphPad Prism5.

### Targeting p-STAT3 by NSC74859 induces autophagy in HNSCC cells

Autophagy and apoptosis often simultaneously occur [14, 15]. Thus, we also examined whether or not NSC74859 induces autophagy in HNSCC cells through morphological and biochemical analyses. Upon autophagy induction, microtubule-associated protein light chain 3 (LC3) can specifically target autophagic membranes to form autophagosomes [12]. To monitor autophagosome formation, we constructed a CAL27 cell line stably expressing the GFP-LC3 fusion gene and used a fluorescent microscope to detect GFP-LC3 punctate dot. As shown in Figure 2A, NSC74859 exposure led to an obvious punctate pattern of LC3II immunofluorescence staining in CAL27 cells compared with the negative controls. The results of fluorescent microscopy showed that the formation of GFP-LC3-labeled vacuoles increased; consistently, the results of Western blot demonstrated the dose-dependent conversion of LC3I to LC3II. Two other well-established autophagy markers were validated in NSC74859-treated cells through Western blot analysis: enhancement of Beclin1, a component of the phosphoinositide 3-kinase (PI3K) complex essential for autophagosome formation [16]; degradation of p62, a link between LC3 and ubiquitinated substrates [17] (Figure 2B).

**Figure 2:** Targeting STAT3 by NSC74859 induced autophagy in HNSCC cells **A.** CAL27 cells transfected with GFP-LC3 plasmid were treated with different concentration of NSC74859 for 24 h. The formation of GFP-LC3 puncta were examined using immunofluorescence and quantified. *Scale bar* 50 μm; **P < 0.01; **B.** CAL27 cells were treated with different concentration of NSC74859 for 24 h, then detected autophagy-associate protein LC3I/II, p62, and Beclin1 by western blot analysis; Densitometric values were quantified using the Image J software, and the data were presented as means ± SEM of three independent experiments. *P < 0.05, **P < 0.01; **C.** CAL27 cells were treated with 100 μM of NSC74859 in the absence or presence of 20 nM Bafilomycin A1 for 24 h, then formation of GFP-LC3 puncta were examined using immunofluorescence and quantified, *P < 0.05, **P < 0.01 *versus* the control group, One-way ANOVA with post-Dunett analysis was used by GraphPad Prism5; ^##^*P* < 0.01 *versus* the NCS74859 (100 μM) group, One-way ANOVA with post-Tukey analysis was used by GraphPad Prism5; **D.** CAL27 cells were treated with 100 μM of NSC74859 in the absence or presence of 20 nM Bafilomycin A1 for 24 h, then the expression of LC3II was quantified by normalization of their densitometry to GAPDH; Densitometric values were quantified using the Image J software, and the data were presented as means ± SEM of three independent experiments. *P < 0.05, **P < 0.01 *versus* the control group, One-way ANOVA with post-Dunett analysis was used by GraphPad Prism5; ^##^*P* < 0.01 *versus* the NCS74859 (100 μM) group, One-way ANOVA with post-Tukey analysis was used by GraphPad Prism5.

Autophagy is a dynamic process of flux; thus, the increased levels of autophagosomes can signify either the induction of autophagy or the blockage of the downstream lysosomal processing of these autophagosomes, or both [18]. Bafilomycin A1 (Baf A1), a specific inhibitor of the vacuolar-type H^+^-ATPase, prevents autophagy at a late stage by inhibiting the fusion between autophagosomes and lysosomes. To monitor autophagic flux, we measured the levels of LC3II and GFP-LC3-positive autophagosomes in the absence or presence of Baf A1. We found that a Baf A1 challenge increased the level of GFP–LC3-positive autophagosomes (Figure 2C) and LC3II in CAL27 cells treated with 100 μM NSC74859 (Figure 2D). The above experiment was repeated in the FaDu cell line and yielded consistent results (Supplementary Figure S3). These results demonstrated that NSC74859 treatment induced autophagic flux in human HNSCC cells *in vitro*.

### Autophagy alleviates NSC74859-induced apoptosis in HNSCC cells

Autophagy may serve as a pro-survival or pro-death mechanism in different cellular contexts [18–21]. 3-MA, a phosphoinositide 3-kinase inhibitor which prevents the induction of autophagosomes to inhibit autophagy flux, was employed to elucidate the mechanism by which autophagy acts in our system [22]. Compared with CAL27 cells that incubated with NSC74859 alone, Pretreatment with 3-MA obviously decreased LC3II but increased cleaved PARP expression, indicating an elevated apoptosis process compared with NSC74859 treatment alone (Figure 3A). Moreover, Annexin V-FITC/PI staining showed that pretreatment of CAL27 cells with 3-MA induced a higher percentage of apoptotic cells (Figure 3B) when compared with NSC74859-treated alone, whereas cells treatment with 3-MA alone showed limited apoptosis-inducing effects on CAL27 cells. To monitor autophagic flux, we also measured the levels of LC3II and cleaved PARP in the absence or presence of CQ. We found that a CQ challenge increases the level of LC3II and cleaved PARP in CAL27 cells treated with 100 μM NSC74859 (Figure 3C). Moreover, Annexin V-FITC/PI staining showed that pretreatment of CAL27 cells with CQ increased the number of apoptotic cells (Figure 3D).

**Figure 3:** Autophagy alleviates NSC74859-induced apoptosis in HNSCC cells CAL27 cells were pretreated with 2 mM 3-MA and incubated with 100 μM NSC74859 for another 24 h. The LC3 and Cl-PARP level **A.** the percentage of Annexin V-positive apoptotic cells **B.** were determined; CAL27 cells were pretreated with 10 μM CQ and incubated with 100 μM NSC74859 for another 24 h. The LC3 and Cl-PARP level **C.** and the percentage of Annexin V-positive apoptotic cells **D.** were determined; **E.** CAL27 cells were treated with DN-ATG5^K130R^ for *ATG5* incubated with 100 μM NSC74859 for another 24 h. The LC3 and Cl-PARP level and the percentage of Annexin V-positive apoptotic cells were determined **F.** GAPDH was the internal standard for protein loading. The values were presented as the means ± SEM. *P < 0.05, **P < 0.01 *versus* the control group, One-way ANOVA with post-Dunett analysis was used by GraphPad Prism5, ^##^*P* < 0.01 *versus* the NCS74859 (100 μM) group, One-way ANOVA with post-Tukey analysis was used by GraphPad Prism5.

Pharmacological inhibitors of autophagy may exhibit autophagy-independent actions [15]. To verify the pro-survival action of autophagy, the effects of NSC74859 were examined in cells in which autophagy-related gene 5 (Atg5), an essential protein for autophagosome formation [23], was downregulated by the transient transfection of dominant negative Atg5 (DN-Atg5^K130R^), which inhibits Atg12 conjugation and autophagosome formation [24, 25]. As shown in Figure 3E, transient transfection of DN-Atg5^K130R^ into CAL27 cells lowered LC3II level but increased cleaved PARP level after NSC74859 treatment compared with that in vector control. This result correlated with the obviously decreased expression of the Atg5-Atg12 complex as detected by Western blot analysis. In addition, flow cytometry showed that the population of Annexin V+FITC/PI− cells remarkably increased (Figure 3F). Our results indicate that STAT3-blockade-induced autophagy serves a pro-survival function in HNSCC cells.

### Akt/mTOR and Erk signaling pathways are involved in NSC74859-induced autophagy in HNSCC cells

In the current study, we detected whether or not Akt/mTOR is involved in NSC74859-induced autophagy by evaluating the levels of p-Akt^S473^ and p-mTOR^S2448^ in CAL27 cells. After incubation with NSC74859 at indicated concentration, Western blot analysis showed that NSC74859 decreased the levels of p-Akt^S473^ and p-mTOR^S2448^. Furthermore, p-S6^S235/236^ as the downstream substrate of mTOR was significantly decreased (Figure 4A). To further investigate the role of Akt/mTOR signaling in autophagy induced by NSC74859, a plasmid expressing the myristoylated and constitutively active form of the Akt1 protein (Myr-Akt) was applied [26]. As expected, over-expression of activated Akt can alleviate NSC74859-induced autophagy (Figure 4B). Several studies reported that the Erk signaling cascade stimulates autophagy by interacting with LC3 [27, 28]. However, whether and how the Erk cascade regulates autophagy remains unknown. In the present study, the level of p-Erk1/2^T202/204^ dose- and time-dependently increased in CAL27 cells treated with different concentration of NSC74859 for 24 h (Figure 4C) or with 100 μM NSC74859 for 6, 12, and 24 h (Figure 4D). To further investigate the role of Erk in autophagy induced by NSC74859, the Erk inhibitor U0126 was employed to block the phosphorylation of Erk1/2. The levels of LC3-II and p-Erk1/2^T202/204^ decreased in CAL27 cells, indicating that autophagy was suppressed by inhibiting p-Erk1/2^T202/204^ expression (Figure 4E). These results suggested that NSC74859 increases autophagy by inhibiting p-mTOR^S2448^ and increasing p-Erk1/2^T202/204^.

**Figure 4:** The Akt/mTOR and Erk signaling pathway are involved in NSC74859-induced autophagy in HNSCC cells **A.** CAL27 cells were treated with different concentration of NSC74859 for 24 h, the level of Akt, *p*-Akt^S473^, mTOR, *p*-mTOR^S2448^, S6 and *p*-S6^S236/236^ were analyzed by western blot in left part. Relative quantitative data were calculated by Image J in the right part; **B.** Western blotting of NSC74859-induced autophagy following the overexpression of a constitutively active form of Akt (Myr-Akt). Cells were transfected with an Akt overexpression (Myr-Akt) or empty vector (pcDNA3) plasmid for 24 hours and then treated with 100 μM of NSC74859 for 24 hours. Levels of Akt, *p*-Akt^S473^, and LC3I/II were measured by western blotting. **C.** CAL27 cells were treated with different concentration of NSC74859 for 24 h, the level of Erk 1/2 and *p*-Erk 1/2^T202/204^ were analyzed by western blot in left part; Relative quantitative data were calculated by Image J in the right part; **D.** CAL27 cells were treated with100 μM of NSC74859 for 6, 12 and 24 h, then western blot was performed to analyze the protein Erk 1/2 and *p*-Erk 1/2^T202/204^; Relative quantitative data were calculated by Image J in the right part; **E.** CAL27 cells were treated with 100 μM of NSC74859 in the presence or absence of the Erk phosphorylation inhibitor U0126 (20 μM) for 24 h. The level of LC3I/II, Erk 1/2 and *p*-Erk 1/2^T202/204^ were determined by western blot analysis in left part. Relative quantitative data were calculated by Image J in the right part. *P < 0.05, **P < 0.01 *versus* the control group, One-way ANOVA with post-Dunett analysis was used by GraphPad Prism5, ^#^*P* < 0.05 *versus* the NCS74859 (100 μM) group, One-way ANOVA with post-Tukey analysis was used by GraphPad Prism5.

### Targeting autophagy and STAT3 signaling blocks tumor growth *in vivo*

Based on the *in vitro* findings, we investigated whether or not the autophagy inhibitor CQ can enhance the antitumor effect of NSC74859 *in vivo*. A xenograft tumor model was established by the subcutaneous inoculation of CAL27 cells into nude mice. Throughout the course of treatment, NSC 74859 (5 mg/kg body weight) did not cause visible side effects or change in body weight of the mice. The antitumor ability of NSC74859 combined with CQ was stronger than that of NSC74859 alone; this combination treatment decreased tumor size and weight (Figures 5A and 5B). Immunohistochemical results revealed that the combination of NSC74859 and CQ decreased p-STAT3^T705^ and Bcl2 expression but enhanced LC3 conversion and p62 expression in the CAL27 xenografts compared with NSC74859 alone (Figure 5C). Meanwhile, Western blot analysis showed that the levels of cleaved PARP and cleaved caspase3 increased with increasing LC3 (Figures 5D and 5E). These data indicated that targeting autophagy and STAT3 signaling reduced the tumor volume and growth rate of HNSCC cells *in vivo*.

**Figure 5:** Targeting autophagy and STAT3 signaling blocks tumor growth *in vivo* **A.** Tumor growth curve of control (vehicle treated) mice, CQ-treated (250 mg/kg body weight) mice, NSC74859-treated (5 mg/kg body weight) mice and co-treatment with CQ (250 mg/kg body weight) and NSC74859 (5 mg/kg body weight) mice. Data represent the mean ± SEM of five mice in each group. **P < 0.01 *versus* the control group, ^#^*P* < 0.05 *versus* the NCS74859 (5 mg/kg body weight) group by the Student *t* test. **B.** Dissected tumor was weighted. **P < 0.01 *versus* the control group, ^#^*P* < 0.05 *versus* the NCS74859 (5 mg/kg body weight) group by the Student *t* test. **C.** Representative images of immunohistochemical analysis of *p*-STAT3^T705^, LC3, Bcl-2 and p62 in tumors. **D.** Western blots of *p*-STAT3^T705^, LC3, Cleaved-Caspase 3 (Cl-Casp 3) and cleaved-PARP (Cl-PARP) in tumor tissues. GAPDH was probed as the loading control. Densitometric values were quantified using the Image J software, and the data were presented as means ± SEM of three independent experiments. *P < 0.05, ** *P* < 0.01 *versus* the control group, one-way ANOVA with post-Dunett analysis was used by GraphPad Prism5; ^##^*P* < 0.01 *versus* the NCS74859 (100 μM) group, One-way ANOVA with post-Tukey analysis was used by GraphPad Prism5.

### Increased p-STAT3^T705^ expression correlates with LC3, LAMP2, and p-Erk1/2 in human HNSCC tissue

Immunohistochemistry for p-STAT3^T705^ was performed on 57 HNSCC tissues and 10 normal oral mucosa tissues to determine whether or not p-STAT3^T705^ expression is linked to HNSCC in human. Compared with normal oral mucosa samples, human HNSCC tissues had significantly higher p-STAT3^T705^ expression in the nucleus (Figure 6A). Using hierarchical clustering analysis, the relationships of p-STAT3, LC3, LAMP2 and p-Erk1/2 in HNSCC were displayed in a visual image. Of interest, the expression of p-STAT3, LC3, LAMP2 and p-Erk1/2 in most of the HNSCC cases (cluster 2) were distinct from normal mucosa (cluster 1), reflecting the significant differences in p-STAT3, LC3, LAMP2 and p-Erk1/2 staining in HNSCC (Figure 6C). Clustering analyses of immunohistochemistry of HNSCC and normal oral mucosa tissues showed that p-STAT3^T705^ expression positively correlated with LAMP2 (*P* = 0.0003, *r* = 0.4315) and p-Erk1/2^T202/204^ (*P* = 0.0055, *r* = 0.3408) but negatively correlated with the autophagic marker LC3 (*P* = 0.0340, *r* = −0.2634) (Figure 6B). These observations are consistent with other reports [5, 29] and suggest that HNSCC tumor cells frequently produce high levels of p-STAT3.

**Figure 6:** Increased p-STAT3^T705^ expression correlates with LC3, LAMP2, and p-Erk1/2 in human HNSCC tissue **A.** Representative immunohistochemical staining (IHC) of p-STAT3^T705^, LC3, LAMP2, p-Erk1/2^T202/204^ in human oral cancer tissue (right) as compared with normal oral mucosa (left) (*Scale bars* = 50 μm); **B.** *p*-STAT3^T705^ was found to be closely associated the LC3 (*P* = 0.0340, *r* = −0.2634), LAMP2 (*P* = 0.0003, *r* = 0.4315) and *p*-Erk1/2^T202/204^ (*P* = 0.0055, *r* = 0.3408); **C.** Hierarchical clustering presented the protein expression correlation of *p*-STAT3^T705^, LC3, LAMP2 and *p*-Erk1/2^T202/204^ in human HNSCC tissue array.

## DISCUSSION

In this study, we conducted *in vitro* and *in vivo* experiments to determine whether or not p-STAT3^T705^ blockade using NSC74859 could induce HNSCC cell death and autophagy. Pharmacological or genetic inhibition of autophagy sensitized HNSCC cells to NSC74859-induced apoptosis. Evidence from a xenograft model proved that suppressing STAT3 activity and inhibiting autophagy can promote tumor regression better than using either treatment alone. These results indicate that autophagy plays a pro-survival role in NSC74859-induced cell death in HNSCC cells. In particular, NSC74859-induced autophagy through blockade of STAT3 signaling pathway is correlated with the Akt/mTOR and Erk pathways.

STAT3 is a transcription factor that can be activated by IL-6, EGF, and other cytokines [30]. STAT3 plays a key role in various biological processes, including inflammation, cell proliferation, migration, survival, and metabolic disorders [31]. Subsequently, the potential oncogenic role of STAT3 was established because constitutive STAT3 activation has been detected in nearly 70% of human epithelial malignancies and hematopoietic malignancies, where increased STAT3 expression is commonly associated with a poor clinical prognosis [4, 30, 32]. In the present study, immunohistochemical analysis of HNSCC and normal oral mucosa tissues verified that p-STAT3 expression was dramatically increased in human HNSCC tissues. These observations are consistent with other reports [5, 29] and suggest that HNSCC tumor cells frequently produce high levels of p-STAT3.

STAT3 is an attractive therapeutic target because its development and regulation display an oncogenic phenotype [5, 33]. Sen et al. found that the JAK kinase inhibitor AZD1480 abrogates STAT3 activation and head and neck squamous cell carcinoma tumor growth [34]. Peyser et al. reported that PTPRT is frequently hypermethylated in HNSCC and PTPRT promoter and methylation is significantly associated with sensitivity to STAT3 inhibition in HNSCC cells [35]. Study by Bonner et al. suggested that head and neck cancer cells were more sensitive to cetuximab after the inhibition of STAT-3 by an inhibiting short hairpin RNA (shRNA) knockdown approach [36]. Sen et al. [37] generated a double-stranded STAT3 oligonucleotide decoy and conducted a clinical trial in head and neck tumors. However, the results of initial clinical trials that utilized STAT3 inhibitors are unsatisfactory. Blocking p-STAT3 potently stimulates the autophagic flux [11]. However, whether or not autophagy promotes cell death or enhances survival remains controversial. Drug-induced autophagy of tumor cells has been reported [38, 39], but most studies support the survival role of autophagy in chemotherapy-induced cell death [40, 41]. Therefore, the potential cause of treatment failure in these settings may be the pro-survival role of autophagy induced by STAT3 inhibitors. Considering that the pharmacological or genetic inhibition of autophagy promotes NSC74859-induced apoptosis, we speculated that NSC74859-mediated autophagy is a pro-survival mechanism rather than a pro-death mechanism. These observations are consistent with other reports [42]. A xenograft tumor model was established by the subcutaneous inoculation of CAL27 cells into nude mice treated with both NSC74859 and CQ. Co-treatment reduced tumor volume compared with NSC74859 alone, indicating that blocking the autophagic flux can enhance the efficacy of NSC74859 on HNSCC cells.

Possible proteins involved were detected in xenografts and HNSCC cells through Western blot and immunohistochemistry to further explore the mechanism by which targeting STAT3 triggers cell death and autophagy, as well as to elucidate the role of p-STAT3^T705^ in each process. At least 30 autophagy-related genes have been identified [43]. *mTOR* is an autophagy-related gene that negatively modulates autophagosome formation in eukaryotic cells [44]. In the present research, we evaluated the level of phosphorylated mTOR to detect whether or not mTOR is involved in NSC74859-induced autophagy. NSC74859 treatment decreased the phosphorylation levels of Akt and mTOR as well as the phosphorylation substrates of mTOR (p-S6^S235/236^) in CAL27 cells. This result indicates that the Akt/mTOR signaling pathway is involved in NSC74859-induced autophagy in CAL27 cells. The Erk signaling cascade plays a key role in autophagy regulation [45, 46]. However, the mechanism underlying this regulation process has yet to be elucidated. The present results verified the importance of Erk activation in NSC74859-induced autophagy. The level of p-Erk1/2^T202/204^ increased in CAL 27 cells treated with different concentration of NSC74859 for 24 h. The Erk phosphorylation inhibitor U0126 was employed to further confirm the role of Erk1/2 in NSC74859-induced autophagy [47]. Treatment with 100 μM NSC74859 and 20 μM U0126 for 24 h decreased the levels of LC3II and p-Erk1/2^T202/204^ in CAL27 cells. This result suggests that autophagic flux can be suppressed by inhibiting the phosphorylation of Erk1/2.

Overall, the present study proved that inhibiting STAT3 signaling by NSC74859 could induce autophagy and apoptosis in HNSCC cells *in vitro* and *in vivo*, and that autophagy induced by NSC74859 plays a pro-survival role. Pharmacological or genetic inhibition of autophagy sensitized HNSCC cells to NSC74859-induced apoptosis. Moreover, the Akt/mTOR and Erk pathways were involved in NSC74859-induced autophagy in HNSCC cells. This interaction may provide significant benefits to HNSCC patients, particularly in combination with other anti-STAT3 agents, because STAT3 has diverse functions and is almost universally activated in HNSCC cancer cells. Therefore, suppressing autophagy can enhance the efficacy of STAT3 signaling blockage on HNSCC cells, and this process might be a promising therapeutic strategy for HNSCC.

## MATERIALS AND METHODS

### Drugs and reagents

NSC74859 was purchased from Selleck (Houston, TX). Bafilomycin A1, 3-Methyladenine (3-MA) and Chloroquine (CQ) was obtained from Sigma (St. Louis, MO). U0126 was obtained from Cell Signaling Technology (Danvers, MA). Lipofectamine 2000 was bought from Invitrogen (Carlsbad, CA). Stock solutions were prepared in dimethyl sulfoxide (DMSO), stored at − 20°C, and diluted in fresh medium for each experiment. The final concentration of DMSO did not exceed 0.1% in any of the experiments to prevent toxicity to cells. The expression vectors encoding dominant negative Atg5 mutant (pCIneo-DN-Atg5K130R), as well as the corresponding empty vectors (pCI-neo) were provided by Prof. Tamotsu Yoshimori (National Institute for Basic Biology, Okazaki, Japan) [25].

### Cell lines

Human HNSCC cell lines CAL27 and FaDu were bought from the American Type Culture Collection (Manassas, VA). Cells were grown in DMEM (Gibco, Carlsbad, CA) with 10% fetal bovine serum (FBS; Gibco) [48]. All cells were grown in a humidified atmosphere of 95% air 5% CO_2_ at 37°C and experiments were performed on 4th and 5th passages generated from the frozen stock.

### Nuclear morphology assessment by Hoechst 33258 staining

CAL27 cells were plated in 24-well tissue culture plates for 24 h and incubated with different concentration of NSC74859 (0 to 200 μM) for 24 h with detailed procedure as previous described [48].

### Apoptosis assay

Apoptosis was quantified with an Annexin V-FITC apoptosis detection kit (BD Biosciences, San Diego, CA, USA) following the manufacturer's instructions as previous described [49].

### GFP-LC3 analysis

CAL27 cells stably expressing GFP-LC3 were obtained by transfecting the cells with EGFP-LC3 plasmid and selected with G418. Transfection using Lipofectamine 2000 Reagent was carried out according to the manufacturer's protocol. After transfection, cells were washed twice with phosphate-buffered saline (PBS), and fresh DMEM was added for further incubation. The formation of GFP-LC3 punctate structures was examined as previously described [50]. The images were photographed using a fluorescence microscope (Leica, Brunswick, Germany).

### Animal studies

All proposals were approved and supervised by the institutional animal care and use committee of Wuhan University [51]. Institutional guidelines for the proper and humane use of animals in research were followed. Female BALB/c nude mice (18–20 g) with 6–8 weeks of age were housing in the Experimental Animal Center of Wuhan University in pressurized ventilated cages according to institutional regulations. CAL27 cells (2 × 10^6^ in 0.2 mL of medium) were inoculated subcutaneously into the flank of the mice. After 14 days, tumor-bearing mice were randomly divided into four groups. Treatment with NSC74859 or CQ or both of them was started 14 days after inoculation of the cells. The experimental group (*n* = 5) was treated with i.p. injections of NSC74859 (5 mg/kg body weight) for 21 consecutive days until the mice were killed, whereas the control group (*n* = 5) received equal volume of PBS only. For CQ and NSC74859 co-treatment experiment, the experimental group (*n* = 5) was treated with i.p. injections of NSC74859 (5 mg/kg body weight) and CQ (250 mg/kg body weight) for 21 consecutive days until the mice were killed, whereas the control group (*n* = 5) received CQ (250 mg/kg body weight) only. Throughout the course of treatment, the mice were monitored daily for any discomfort and weighed every other day to check for physical condition. Tumor volumes were calculated to determine the tumor growth according to the formula (width^2^ × length)/2 as previous described [49].

### Western blot analysis

Western blot analysis were performed as previously described with details in Supplementary Material and Methods [48].

### Human HNSCC tissue microarray

Human HNSCC tissue microarray HN803a including 57 confirmed paraffin-embedded HNSCC and 10 normal oral mucosa specimens were obtained from US Biomax with detailed clinical and pathological information as previous describe [52].

### Immunohistochemistry, hierarchical clustering and data visualization

Immunohistochemistry (IHC) and hierarchical clustering were performed as described previously [53]. Firstly, immunohistochemical analyses of human tumor samples were converted into scaled values centered at zero in Microsoft Excel, then the Pearson's correlation coefficient was carried out with Cluster 3.0 with average linkage to achieve the hierarchical analysis results were visualized using the Java Tree View 1.1.6 version. Finally, the clustered data were arranged with markers on the horizontal axis and tissue samples on the vertical axis. Biomarkers with a close relationship are located next to each other.

### Statistical analysis

All the data were presented as mean ± SEM. Data were analyzed and visualized using Graph-Pad Prism 5.0. One-way analysis of variance followed by post Tukey Test were used to determine statistical differences between treatment groups. All experiments were independently repeated in triplicate. *P* < 0.05 was regarded as statistical significance; all tests were two-sided and no corrections were applied for multiple significance testing. * or ^#^, ** or ^##^, and *** indicated *P* < 0.05, *P* < 0.01 and *P* < 0.001, respectively.

## SUPPLEMENTARY MATERIALS, METHODS AND FIGURES


